# Despite Blocking Doxorubicin-Induced Vascular Damage, Quercetin Ameliorates Its Antibreast Cancer Activity

**DOI:** 10.1155/2020/8157640

**Published:** 2020-08-07

**Authors:** Hanan A. Henidi, Fahad A. Al-Abbasi, Mohamed A. El-Moselhy, Hany M. El-Bassossy, Ahmed M. Al-Abd

**Affiliations:** ^1^Research Department, Health Sciences Research Center, Princess Nourah Bint Abdul Rahman University, Riyadh 13412, Saudi Arabia; ^2^Department of Biochemistry, Faculty of Science, King Abdulaziz University, Jeddah 21589, Saudi Arabia; ^3^Department of Clinical Pharmacy and Pharmacology, Ibn Sina National College for Medical Studies, Jeddah 22421, Saudi Arabia; ^4^Department of Pharmacology and Toxicology, Faculty of Pharmacy, Zagazig University, Zagazig 44519, Egypt; ^5^Department of Pharmaceutical Sciences, College of Pharmacy & Thumbay Research Institute for Precision Medicine, Gulf Medical University, Ajman 4184, UAE; ^6^Department of Pharmacology, Medical Division, National Research Centre, Cairo 12622, Egypt

## Abstract

Quercetin is a naturally occurring flavonol present in many foods. Doxorubicin is an effective anticancer agent despite its dose-limiting cardiovascular toxicity. Herein, we investigated the potential protective effects of quercetin against doxorubicin-induced vascular toxicity and its effect on the therapeutic cytotoxic profile of doxorubicin in breast cancer cell lines. The incubation of isolated aortic rings with doxorubicin produced concentration-dependent exaggeration of vasoconstriction responses to phenylephrine but impaired vasodilation responses to acetylcholine. Coincubation with quercetin completely blocked the exaggerated vasoconstriction responses and the impaired vasodilation. In addition, doxorubicin incubation increased reactive oxygen species generation from the isolated aorta, while coincubation with quercetin inhibited ROS generation back to normal values. On the other hand, quercetin in combination with doxorubicin, doubled the IC_50_ of doxorubicin alone in MCF-7 cells from 0.4 ± 0.03 to 0.8 ± 0.06 *μ*M. To a lesser extent, the IC_50_ of doxorubicin did not change after combination with quercetin in MDA-MB-231 cells. These findings indicate a significant antagonistic interaction between quercetin and doxorubicin in the aforementioned cell lines. Only in T47D cells, quercetin combination with doxorubicin was an additive interaction (CI − value = 1.17). Yet, quercetin significantly impaired the immediate phase of intracellular ROS generation by doxorubicin within breast cancer cells from 125.2 ± 3.6% to 102.5 ± 3.9% of control cells. Using annexin-V/FITC staining technique, the quercetin/doxorubicin combination showed a significantly lower percent of apoptotic cells compared to doxorubicin alone treated cells. Cell cycle distribution in breast cancer cells was performed using DNA content flowcytometry after propidium iodide staining. Quercetin induced significant accumulation of cells in the S phase as well as in the G_2_/M phase within both MCF-7 and MDA-MB-231 cell lines and interfered with doxorubicin-induced cell cycle effects. Interestingly, quercetin was found to inhibit the P-glycoprotein ATPase subunit with a consequent enhanced intracellular concentration of doxorubicin in MDA-MB-231 and T47D cells. In conclusion, quercetin, despite its potent vascular protective activity against doxorubicin, was found to influence doxorubicin-induced antibreast cancer effects via pharmacodynamic as well as cellular pharmacokinetic aspects.

## 1. Introduction

Doxorubicin (DOX) is one of the primary anthracycline antibiotics that have been successfully and efficiently used as an anticancer agent since the 1970s. DOX is often used in the treating of breast cancers, ovarian cancers, and other types of carcinoma [1, 2]. A significant restriction imposed on the usage of DOX is its cardiotoxicity, with the total cumulative dose being the only criteria used for prediction [3]. Doxorubicin's high affinity to iron leads to the formation of a complex that increases free radical production and further induces oxidative damage. Cardiomyocytes are more prone to oxidative damage due to their limited potential of regeneration and their lack of necessary oxidative stress enzymes that scavenge hydrogen peroxide and other reactive oxygen species (ROS) [4]. Doxorubicin-induced cardiotoxicity can be prevented by balancing the intracardiac generated ROS with powerful antioxidants and particularly of natural origin. Apart from its toxic effects, DOX may also cause endothelial damage, which contributes to vascular toxicity and other side effects. A couple of studies show that superoxide dismutase and similar antioxidant enzymes are significantly involved in the meditation of oxidative stress and significantly decrease the detrimental effects of DOX on vascular function [5, 6].

Natural medicine in the field of cancer treatment is drawing major attention of researchers in the drug discovery field [7]. Nonetheless, utilizing naturally derived compounds as adjuvant agents are used to improve the activity of well-known chemotherapeutics [8]. Several chemical families and plant-derived bioactive compounds showed significant and promising chemotherapeutics as well as chemomodulatory anticancer effects [9–11]. Flavonoids are naturally occurring polyphenolic potent antioxidants abundant in several edible vegetables and fruits. Their inherent safety makes them attractive candidates for reducing the exacerbation of cardiotoxicity attributed to conventional anticancer drugs such as anthracyclines [12–14]. Quercetin, a polyphenolic compound found in several fruits and vegetables, possesses antioxidant, anti-inflammatory, and antibiotic activities [15]. Previous researches suggest that quercetin has various benefits for different cell types such as myocytes, hepatocytes, gonadal cells, and renal tubular cells and particularly in ischemia/reperfusion tissue injuries. Within the flavonoid family, quercetin is a suprapotent ROS scavenger, not to mention superoxide anion, singlet oxygens, lipid peroxy free radicals, and copper-catalyzed oxidation [16]. Reports suggest that quercetin can scavenge ROS and inhibit the activation of the ERK/MAP-kinase pathway in ROS-induced cardiomyopathy [17, 18].

In our previous studies, quercetin had the potential to increase the cardioprotective effects of lostran against chronic DOX cardiotoxicity through its antioxidant and anti-inflammatory properties [19]. At the vascular level, quercetin has the potential to prevent diabetes-based vascular complications in both insulin deficiency and insulin-resistant conditions through inhibiting several inflammatory pathways [20]. Herein, we examined the potential vascular protective effects of quercetin against DOX-induced acute vascular injury, with a reciprocal glance towards its influence on DOX anti breast cancer properties.

## 2. Materials and Methods

### 2.1. Chemicals

Dulbecco's modified eagle medium (DMEM), RPMI-1640 medium, heat-inactivated fetal bovine serum (FBS), Trypsin-EDTA (0.25%), and penicillin-streptomycin-glutamine were procured from Thermo Fisher Scientific, Gibco (Waltham, MA, USA). Doxorubicin, aetylecholine, phenylephrine, quercetin (purity > 95% by HPLC method; Cat Q4951), dimethyl sulfoxide (DMSO), and other chemicals were procured from Sigma-Aldrich (St Louise, MO, USA). Annexin V-FITC apoptosis detection kit was obtained from Abcam Inc., Cambridge Science Park, Cambridge, UK.

### 2.2. Assessing the Protective Effect of Quercetin against Doxorubicin-Induced Vascular Damage

#### 2.2.1. Animals and Aortic Ring Preparation

Male Wistar rats (King Abdul-Aziz University, Jeddah, Saudi Arabia) weighing 150-200 g, aged 6 weeks were maintained under controlled room conditions and provided with standard food pellets and water *ad libitum*. Animals were sacrificed by cervical dislocation followed by exsanguination. Thoracic aortae were isolated as described in our previous publications. Isolated aortae were sectioned into 3 mm long rings and incubated within the organ bath with doxorubicin (10 *μ*M) with or without different concentrations of quercetin (10–300 *μ*M) for one hour before assessing their vasoconstriction properties. Experimental procedures and animal handling were done according to the Saudi Arabia Research Bioethics and Regulations [21].

#### 2.2.2. Vascular Reactivity

Vascular reactivity of the isolated thoracic aorta rings was performed using the previously detailed isolated artery technique [22]. Surgically isolated aortic rings were suspended in organ baths containing Krebs-Hensleit buffer solution under constant tension (1500 mg) at 37°C and gassed with 95% O2/5%CO2 (carbogen) for 60 min. To examine the vasoconstrictive response of the isolated aortic rings, cumulative concentrations (10^−9^ to 10^−5^ M) of phenylephrine (PE) were obtained and expressed as milligram tension with/without DOX, quercetin, and their combination. Prior to assessing relaxant responses, rings were precontracted with submaximal concentrations of PE (10^−6.5^M to 10^−5.5^M). Additional cumulative concentrations of acetylcholine (Ach, 10^−9^ to 10^−5^ M) were added to the organ bath in order to assess the concentration-dependent relaxation responses with/without DOX, quercetin, and their combination. Responses were recorded as a percentage of PE precontraction tension. Vasodilation/vasoconstrictive responses were recorded by isometric force transducers connected to a data acquisition system (PowerLab®, ADInstruments, Australia) running LabChart® software (ADInstruments, Australia). Control groups were exposed to drug-free media. Optimum DOX concentrations were determined after pilot dose response effects and as per our previous publication [10].

#### 2.2.3. Vascular Oxidative Stress

Basal levels of ROS within aortic rings were measured according to the method of Ahmed et al. with minor modifications [21]. Before assessing ROS generation, aortic rings were first preincubated with doxorubicin (10 *μ*M) with or without quercetin (10 and 100 *μ*M) in the Krebs–Henseleit buffer for 45 min. Following that, the aortic tissues were incubated in 10 *μ*M 2,7-dichlorodihydrofluorescein diacetate (DCFH-DA) plus 0.1% pluronic F-127 for 30 min at 37°C in the dark. Then, the fluorescence of DCFH-DA was measured at *λ*_ex/em_ of 485 nm/515 nm, and parallel background fluorescence caused by buffer solution and unconverted DCFH was used to correct the DCFH-DA fluorescence signal. ROS-induced fluorescence was expressed as fluorescence units per mg protein (F (mg protein)^−1^).

### 2.3. Assessing the Effect of Quercetin on the Cytotoxic Profile of Doxorubicin

#### 2.3.1. Cell Culture

Three different human breast cancer cell lines were used; two human breast adenocarcinoma cell lines (double-negative, MCF-7 and triple-negative, MDA-MB 231) and human ductal carcinoma cell line (T47D) were obtained from Nawah Scientific, Mokkatam, Cairo, Egypt. All cell lines were cultured in their optimum media (DMEM or RPMI-1640 media) with 10% FBS, 100 U/mL penicillin, and 100 *μ*g/mL streptomycin and passaged in a humidified incubator at 37°C with 5% CO2. Cells were passaged at 80-90% confluence by trypsinization based on standard procedures.

#### 2.3.2. Cytotoxicity Assessment

The cytotoxicity of DOX, quercetin, and their combination was assessed using a sulforhodamine B (SRB) assay based on the method of Skehan et al. [23]. Cells were plated in 96-well plates (10^3^ cells/well) and allowed to attach for 24 hours before treatment. Cells were exposed to DOX, quercetin, or their equitoxic combination for 72 h and then fixed by adding 10% (*w*/*v*) trichloroacetic acid (TCA) for 1 h at 4°C, followed by washing with distilled water. Cell were stained with 0.4% (*w*/*v*) SRB for 10 min at room temperature in a dark place and washed with 1% (*v*/*v*) glacial acetic acid, and after the plates were dried, the dye was solubilized by Tris-HCl. Absorbance of viable cells was measured at 540 nm with an ELISA microplate reader and compared to control untreated cells (cells exposed to drug-free media).

#### 2.3.3. Data Analysis

Cell viability and the dose-response curves were calculated by using the *E*_max_ model:

(1) %Cell viability=100−R×1−DmKdm+Dm+R,

where *R* is the resistance fraction, [*D*] is the drug concentration used, *K*_*d*_ is the drug concentration at which 50% of the maximum effect is obtained, and *m* is a Hill-type coefficient. The IC_50_ value represents the concentration of a drug that is needed to inhibit cell growth by half. *R* values represent cell resistance to treatment under investigation and are calculated after fitting to the *E*_max_ model (i.e., *K*_*d*_ = IC_50_ when *R* = 0 and *E*_max_ = 100 − *R*).

The combination index (CI) was calculated from the formula:

(2) $$\begin{array}{c} \text{CI}=\frac{{\text{IC}}_{50}\text{ of drug }\left(x\right)\text{ in combination}}{{\text{IC}}_{50}\text{ of drug }\left(x\right)\text{ alone}}+\frac{{\text{IC}}_{50}\text{ of drug }\left(y\right)\text{ in combination}}{{\text{IC}}_{50}\text{ of drug }\left(y\right)\text{ alone}}. \end{array}$$

The nature of drug interaction is defined as synergism if CI < 0.8, antagonism if CI > 1.2, and additive if CI ranges from 0.8 to 1.2 [24, 25].

#### 2.3.4. Analysis of Cell Cycle Distribution

Cells were treated with the precalculated IC_50_s of drugs or drug-free media (control cells) for 24 hours. After treatment, cells were harvested with trypsin/EDTA, washed twice with ice-cold PBS, and resuspended in 0.5 mL of PBS. Cells were fixed with 60% ice-cold ethanol for a minimum of one hour at 4°C and stored at -20°C. After two washes with PBS, cells resuspended in 1 mL of PBS containing 50 *μ*g/mL RNAase-A and 10 *μ*g/mL propidium iodide (PI) and incubated for 20 min in the dark at room temperature. DNA contents were analyzed by FACSVantage™ (Becton Dickinson Immunocytometry Systems, San Jose, CA, USA). For each sample, 10,000 events were acquired. Cell cycle distribution was calculated using CellQuest software (Becton Dickinson Immunocytometry Systems, San Jose, CA, USA).

#### 2.3.5. Apoptosis Assessment Using Annexin V-FITC Staining Coupled with Flowcytometry

To assess the effect of DOX, quercetin, and their combination on programmed/nonprogrammed cell death, apoptotic and/or necrotic cells were determined using Annexin V-FITC apoptosis detection kit (Abcam Inc., Cambridge Science Park, Cambridge, UK). Briefly, T47D cells were treated with the predetermined IC_50_s; or drug-free media (control cells) for 24 h and collected by trypsinization, washed twice with ice-cold PBS, and resuspended in 0.5 mL of annexin V-FITC/PI solution for 15 min in the dark according to the manufacturer's protocol. After staining at room temperature, cells were injected through ACEA Novocyte™ flowcytometer (ACEA Biosciences Inc., San Diego, CA, USA) and analyzed for FITC and PI fluorescent signals using FL1 and FL2 signal detector, respectively (*λ*_ex/em_ 488/530 nm for FITC and *λ*_ex/em_ 535/617 nm for PI). For each sample, 12,000 events were acquired. Positive FITC and/or PI cells were quantified by quadrant analysis and calculated using ACEA NovoExpress™ software (ACEA Biosciences Inc., San Diego, CA, USA).

#### 2.3.6. Determination of Cellular Reactive Oxygen Species (ROS) Induced by DOX and Its Combination with Quercetin

To explain the antagonistic effect between quercetin and DOX in MCF-7 cells, the short-term and the long-term ROS scavenging activities of quercetin were assayed using a DCFDA cellular ROS detection assay kit (Abcam Inc., Cambridge Science Park, Cambridge, UK) after 1 h and 24 h of exposure to DOX, quercetin, and their combination in comparison to positive and untreated control cells. Exponentially growing cells were collected using 0.25% Trypsin-EDTA and plated in 96-well plates at 5000-10,000 cells/well. Cells were then exposed to test compounds, TBHP (positive control), or drug-free media (control cells) and further incubated for 1 h (immediate phase)/24 h (delayed phase). Total ROS was determined in situ by adding DCFDA solution directly to cells after treatment with test compounds and further incubation for 30 minutes. Intracellular ROS was determined in situ after washing cells twice with ice-cold PBS and incubation with the DCFDA solution for 1 hour more. The fluorescent signal of DCFDA was measured using SpectraMax® multimode microplate reader (Molecular Devices, LLC, Sunnyvale, CA, USA) at *λ*_ex/em_ 495/529 nm. The fluorescent signal was corrected based on cell-free coincubation of DCFDA solution with test compounds. ROS concentrations were then normalized based on the cell count in each sample using the SRB assay. Total ROS scavenging capacity of quercetin represents its overall antioxidant properties while the intracellular ROS scavenging activity represents quercetin antioxidant properties after cellular internalization (uptake).

#### 2.3.7. The Influence of Quercetin on the Cellular Pharmacokinetics of P-Glycoprotein Substrates

To assess the effect of quercetin on cellular pharmacokinetics of P-gp substrates such as DOX, its potential inhibitory effect for the efflux pumping activity of P-gp was assessed using a noncytotoxic fluorescent probe (rhodamine). Herein, the intracellular rhodamine concentration was determined with and without coexposure of cells under investigation to serial concentrations of quercetin and compared to VRP as a standard P-gp inhibitor. Briefly, exponentially proliferating cells were plated in 96-well plates at a plating density of 104 cells/well. Cells were exposed to equimolar concentrations of rhodamine, rhodamine/quercetin, or rhodamine/verapamil for 24 h at 37°C. Subsequently, plates were washed thrice with ice-cold PBS, and rhodamine concentration was measured spectroflourometrically at *λ*_ex/em_ of 482/550 nm. Rhodamine concentrations were normalized based on cell number [11].

#### 2.3.8. Determining Submolecular Interaction Characteristics between P-gp Protein and Quercetin

P-gp inhibitors block its efflux pumping activity via competitive binding to its binding site subunit or inhibiting P-gp ATPase subunit activity. Human recombinant membrane-bound P-gp proteins attached to ATPase subunit (Pgp-Glo™ Assay Systems, Promega Corporation, Madison, WI, USA) was used as described in our previous publications to define the mechanism of P-gp inhibition due to accumulation/consumption of ATP molecules [26]. Briefly, quercetin (10 *μ*M) was incubated with Pgp-Glo™ assay systems as per the manufacturer's protocol. Rates of ATP consumptions were determined by measuring ATP-firefly luciferase system luminescence. Competitive binding to the P-gp substrate binding site subunit results in stimulating ATPase activity and increases ATP consumption, while ATPase inhibitors would decrease the ATPase enzyme activity and decrease ATP consumption rate. Sodium vanadate and verapamil were used as two different positive controls (ATPase inhibitors and binding site blocker, respectively). ATP consumptions were calculated and presented as remaining ATP concentration and normalized per P-gp protein concentration (pmole ATP/*μ*g P-gp protein).

### 2.4. Statistical Analysis

Data are expressed as mean ± SEM using GraphPad prismTM software (GraphPad Software Inc., La Jolla, CA, USA) for Windows version 5.00. Analysis of variance (ANOVA) was used followed by Newman-Keuls' post hoc test.

## 3. Results

### 3.1. Quercetin Protects from DOX-Induced Vascular Toxicity

One hour of incubating the isolated aortic rings with DOX led to a concentration-dependent increase in vasoconstriction responses to phenylephrine (PE) that reached statistical significance at a concentration of 10 *μ*M DOX (*p* < 0.05, Figures 1(a) and 1(c)**)**. Similarly, DOX incubation lead to concentration-dependent impairment in isolated aorta vasodilation responses to acetylcholine that reached statistical significance at a concentration of 10 *μ*M DOX (*p* < 0.05, Figures 1(b)and 1(d)**)**.

Coincubation with quercetin led to concentration-dependent inhibitions of the DOX-induced exaggerated vasoconstriction responses to PE that retains in controlling response values starting from 10 *μ*M quercetin and even below control responses at higher concentrations of quercetin (30-300 *μ*M, *p* < 0.05, Figure 2(a)). In addition, incubation of normal control aorta with quercetin only led to concentration-dependent alleviations of vasoconstriction responses to PE that reached statistical significance only at the highest concentration of quercetin, 300 *μ*M (*p* < 0.05, Figure 2(b)).

Likewise, coincubation with quercetin led to concentration-dependent alleviations of the DOX-induced impairments in the vasodilation responses to acetylcholine that reached statistical significance with 30 *μ*M quercetin and retained to control responses values at quercetin concentrations of 100 and 300 *μ*M (*p* < 0.05, Figure 2(c)). However, incubation of normal control aorta with quercetin did not have a significant effect on the vasodilation responses to acetylcholine (Figure 2(d)).

### 3.2. Quercetin Scavenges Vascular ROS Generated by DOX In Situ

The vascular protective effects of quercetin against DOX-induced vascular damage were further investigated in situ by measuring ROS concentration within aortic tissues. The incubation of isolated aorta with DOX at a concentration of 10 *μ*M for one hour (the same conditions of the vascular reactivity studies above showed a significant increase in basal aortic ROS generation compared with control (*p* < 0.05)). Coincubation with quercetin led to significant inhibition of DOX-induced excessive ROS production that returns to control values at concentration 10 *μ*M of quercetin and even below control values at higher concentration of quercetin, 100 *μ*M (*p* < 0.05, Figure 3**)**.

### 3.3. Cytotoxicity Assessment of Doxorubicin, Quercetin, and Their Combination against Breast Cancer Cell Lines

To identify whether quercetin with its high ROS scavenging capacity would ameliorate DOX cytotoxicity against breast cancer cells, the dose-response curves of DOX, quercetin, and their equitoxic combination were plotted in three different breast cancer cell lines. In the MCF-7 cell line, DOX showed a gradient killing effect with increasing concentration and viability started to drop at 0.3 *μ*M. The calculated IC_50_ for DOX alone was 0.35 ± 0.1 *μ*M quercetin had a much weaker cytotoxic effect with calculated IC_50_ of 97.7 ± 7.2 *μ*M. The equitoxic combination of quercetin with DOX significantly increased DOX IC_50_ to 0.8 ± 0.1 *μ*M (Figure 4(a)) with CI-value of 3.2 (antagonistic interaction) (Table 1).

Similarly, DOX showed a gradual killing effect with increasing concentration in MDA-MB-231 cells. The calculated IC_50_ for DOX alone was 0.8 ± 0.2 *μ*M. Quercetin also had a weaker cytotoxic effect with a calculated IC_50_ of 38.4 ± 4.8 *μ*M. The equitoxic combination of quercetin with DOX did not induce any significant change in the IC_50_ of DOX (Figure 4(b)) with CI value of 2.04 (antagonistic interaction) (Table 1).

In the T47D cell line, the IC_50_s of DOX and quercetin alone were 0.7 ± 0.09 *μ*M and 78.4 ± 11.9 *μ*M, respectively. Equitoxic combination of quercetin with DOX significantly improved the cytotoxic profile of DOX in the T47D cell line decreasing its IC_50_ to 0.36 ± 0.05 *μ*M (Figure 4(c)). The calculated CI value for DOX with quercetin was 0.96, which indicates an additive interaction (Table 1).

In order to explain the antagonistic effect between quercetin and DOX in MCF-7 cells, we further investigated the effect of the quercetin combination with DOX on ROS generation within MCF-7 breast cancer cells after exposure to the predetermined IC_50_s for 1 h (immediate phase) and 24 h (delayed phase) besides measuring its total *in situ* ROS scavenging capacity. Total ROS scavenging capacity of quercetin represents its overall antioxidant properties while the intracellular ROS scavenging activity represents quercetin antioxidant properties after cellular internalization or uptake. DOX significantly increased the immediate phase of intracellular ROS generation from 100 ± 4.4% to 125.2 ± 3.6% compared to control cells (Figure 4(d)). After prolonged exposure, ROS was significantly lower in DOX-treated cells compared to the control (Figure 4(e)). This might be attributed to depleting the intracellular ROS in the interaction with the free intracellular thiol groups. Total ROS (intracellular and extracellular) was significantly higher after DOX treatment compared to the control group (Figure 4(f)). Quercetin significantly ameliorated the immediate effect of DOX in inducing ROS bringing its level back to normal but did not normalize delayed or total ROS generated in response to DOX treatment (Figures 4(d)–4(f)).

### 3.4. Cell Cycle Distribution Analysis of Breast Cancer Cells after Treatment with DOX, Quercetin, and Their Combination

To measure the influence of DOX, quercetin, and their combination on the cell cycle distribution of breast cancer cells, MCF-7, T47D, and MDA-MB-231 cells were treated with the predetermined IC_50_s for 48 h, and DNA content was quantified after PI staining using flow cytometry. In the MCF-7 cell line, quercetin alone did not induce any significant change in the different cell cycle phases despite a marginal decrease in the nonproliferating cell fraction (G_0_/G_1_ phase) from 76.1 ± 0.4% to 69.1 ± 0.7% with a reciprocal marginal increase in the G_2_/M cell population from 11.7 ± 1.6% to 16.3 ± 1.8%. DOX alone induced a significant accumulation of cells in the G_2_/M phase due to significant cell cycle arrest in the S phase populations. However, quercetin combination reverted all DOX-induced cell cycle arrest and brought all cell populations to be nonsignificantly different from normal untreated cells (Figure 5(a)).

In the triple-negative more resistant MDA-MB-231 cell line, quercetin induced a marginal but significant increase in the S phase cell population with a reciprocal decrease in the nonproliferating cell fraction (G_0_/G_1_ phase) from 57.8 ± 1.1% to 51.3 ± 0.81%. In addition, quercetin combination with DOX induced a significant increase in the G_2_/M phase cell population from 34.3 ± 1.4% to 39 ± 0.5% (Figure 5(b)).

In the T47D cell line, DOX induced a significant arrest in the G_2_/M cell fraction from 14.4 ± 2.1% to 28 ± 2% with a reciprocal significant decrease in both G_0_/G_1_ cell population and synthesis phase (S phase population) from 71.5 ± 3% to 62 ± 2.2% and from 9.7 ± 1.4% to 4.7 ± 0.5%, respectively. Like MCF-7 cells, quercetin's combination with DOX completely reverted its cell cycle interference effects back to normal values (Figure 5(c)).

### 3.5. Effect of DOX, Quercetin, and Their Combination on Apoptosis/Necrosis of Breast Cancer Cells

To accurately define and quantify the mechanism of cell death (apoptosis or necrosis) induced by DOX, quercetin, and their combination, T47D cells were stained with annexin-V/FITC and PI followed by flow cytometry after exposure to their predetermined IC_50_s. DOX alone induced significant apoptosis and necrosis after 24 h of exposure compared to the control untreated cells (Figures 6(a), 6(c), and 6(e)). Similarly, but to a lesser extent, quercetin induced significant apoptosis and necrosis in T47D cells after 24 h of exposure (Figures 6(a), 6(b), and 6(e)). Quercetin's combination with DOX significantly decreased apoptotic cells with a reciprocal significant increase in the nonprogrammed necrotic cell death compared to DOX treatment alone (Figures 6(c)–6(e)).

### 3.6. Effect of Quercetin on the Cellular Pharmacokinetics of DOX within Breast Cancer Cells

Quercetin and many naturally occurring polyphenolic/flavonoids are known with their P-glycoprotein efflux pump interference properties. This results in increased intracellular concentration P-gp substrates such as DOX. Herein, the molecular basis of quercetin interaction with the different subunits of the P-gp efflux pump was studied using human recombinant P-gp ATPase unit bound to P-gp substrate binding subunit and compared to two different positive controls (Sod. vanadate and verapamil). Sod. vanadate (positive control P-gp ATPase subunit inhibitor) resulted in increasing the remaining ATP significantly. On the other hand, verapamil (positive control as competitive P-gp substrate binding site inhibitor) stimulates the consumption of ATP resulting in a significant decrease in the remaining ATP concentration. Quercetin was found to inhibit the P-gp ATPase subunit with a resultant increase in the remaining ATP concentration (Figure 7(a)).

Further assessment for quercetin-induced intracellular trapping activity for P-gp fluorescent noncytotoxic substrate (rhodamine) was undertaken on the three breast cancer cell lines under investigation. Quercetin did not induce any significant change in the intracellular concentration of rhodamine at any concentration (up to 100 *μ*M), neither did verapamil in MCF-7 cells (Figure 7(b)). In MDA-MB-231, quercetin and verapamil (P-gp-positive control inhibitor) increased the intracellular concentration of rhodamine only at 100 *μ*M concentration (Figure 7(c)). Entrapment of rhodamine within T47D cells was observed after treatment with quercetin at concentrations as low as 30 *μ*M similar to verapamil (Figure 7(d)).

## 4. Discussion

DOX is one of the most commonly used anticancer agents for the treatment of several malignancies such as hepatocellular carcinoma, leukemia, lymphoma, osteosarcoma, and breast cancer. Yet, DOX results in dose-limiting cardiovascular toxicities due to the formation of ROS within cardiac muscles which limit its clinical use [27]. It is worth mentioning that DOX-induced cytotoxicity is largely attributed to the formation of ROS within tumor cells/tissues. Quercetin is a well-known flavonol with a powerful antioxidant capacity which protects several organs/tissues from oxidative stress damage. In addition, quercetin possesses acceptable bioavailability and pharmacokinetics distribution after oral ingestion of quercetin-rich diets [8]. According to several studies, quercetin protected against DOX-induced cardiotoxicity [19, 28, 29]. Herein, we further studied the potential protective role of quercetin against DOX-induced vascular toxicity while checking the influence of quercetin ROS scavenging ability on DOX-induced cytotoxicity against breast cancer cells.

Two strategies to protect from DOX-induced cardiotoxicity are used; chemical/structural modification and drug combination with cardioprotective agents such as dexrazoxane [30, 31]. In addition, previous preclinical studies confirmed the important role of several natural products in controlling/inhibiting DOX-induced myocardial toxicity due to reduced ROS concentration and augmented the level of antioxidant enzymes [32]. Quercetin significantly protected against doxorubic-induced vascular damage, in terms of restoring normal vascular contraction and relaxation. Our results concur with other studies showing that DOX exposure increased the contractile responses to phenylephrine and other adrenergic agonists and attenuates relaxation to both endothelium-dependent and endothelium-independent vasodilators [10, 33]. In our observation, it was found that DOX-induced vascular dysfunction occurs within one hour of aortic ring exposure to DOX. This could be explained by the direct effects of DOX on Ca^2+^ channels. Kim et al. have reported that Ca^2+^ release begun to increase at approximately 30 min after DOX treatment [34]. Previous studies have been suggested that DOX increases the opening probability of sarcoplasmic reticulum (SR) calcium release channels [35, 36], inhibits Na^+^-Ca^2+^ exchanger [37], or activates L-type cardiac calcium channel [38]. Yet, the elevated intracellular Ca^2+^ concentration can lead to excessive ROS generation [39] and would potentially exacerbate smooth muscle damage and dysfunction. In the current work, the combination of quercetin with DOX significantly decreased the contractile responses of aortic smooth muscles compared to DOX alone. It was found before that intracellular Ca^2+^ release was blocked by the pretreatment with many naturally occurring antioxidants such as *α*-lipoic acid and *α*-tocopherol [40]. In addition, our results showed that DOX resulted in increased ROS generation within the vascular tissues of the aortic rings. On the other hand, quercetin significantly decreased the ROS concentration within aortic tissues compared to DOX-treated tissues.

Despite its vascular protective effects, quercetin ameliorates DOX-induced antibreast cancer properties against MCF-7 and MDA-MB-231 cell lines with profound and moderate antagonistic interaction, respectively. The intracellular ROS release phenomenon is attributed to the unique chemical structure of DOX and anthraquinones in general. In our work, antagonistic interaction between DOX and quercetin is possible to be explained via the rapid (immediate) ROS scavenging ability of quercetin. Intracellular ROS scavenging effect of quercetin might scavenge the intracellular DOX-induced ROS and diminish the intracellular active form DOX. Previous reports explained decreased doxorubicin-induced cardiotoxicity in vitro and in vivo due to quercetin treatment by the reduction of the intracellular oxidative stress [29]. Similarly, Du et al. reported the antagonistic effect of quercetin to DOX against murine breast cancer (4T1) cells [41]. In another study, quercetin did not enhance the cytotoxicity of doxorubicin in MCF-7 and MDA-MB 231 breast cancer cell lines [42]. Quercetin was reported to induce apoptosis in several tumor cell lines [43]. However, MCF-7 is known to be deficient in caspase-3 enzyme with a subsequent disabled apoptosis pathway [25, 44, 45]. This might narrow the possibility for quercetin-induced tumor-killing effect alone and in combination with doxorubicin in MCF-7 cells and might partly explain their significant antagonism. In addition, quercetin-induced antagonism in some breast cancer cells might be attributed to its strong estrogenic activity and hence its proliferative impact on oestrogen receptor-positive breast cancer cells [46]. The antagonistic effects of quercetin towards DOX-induced cytotoxicity were further observed in the form of reverting DOX-induced cell cycle interference as well as DOX-induced apoptotic effect. Similar results could be found in other human tumor cells; however, quercetin aborted DOX-induced apoptosis in normal rat spleen cells and cardiomyocyte cells (H9C2) [28, 41]. Only in T47D cells, the interaction between DOX and quercetin was not antagonistic; however, it was only additive (nonsynergistic). Equitoxic combination enables the utilization of Chou and Talaly mathematical combination index analysis to evaluate the nature of interaction between two cytotoxic/potentially cytotoxic agents [47–49]. We and others have been utilizing this adjusted equitoxic combination analysis for several decades [48, 50, 51]. It is well known that DOX is a P-gp substrate and is highly affected by the expression as well as the activity of P-gp and related efflux proteins [52, 53]. Quercetin and many naturally occurring polyphenolic and flavonoids are known with their P-gp inhibitory effects [54]. Other terpenoids such as bacopaside-I and bacopaside-II inhibit other membrane transport systems (aquaporins) [55].The unique additive interaction between DOX and quercetin in T47D cells could be explained by the inhibitory effect of quercetin to P-gp-associated ATPase subunit and subsequent enhanced intracellular accumulation of DOX. Quercetin-induced intracellular accumulation of the P-gp substrate was observed in T47D at a lower concentration compared to MDA-MB-231 cells. While no accumulation of P-gp substrate was observed in MCF-7 cells. The expression of P-gp and related efflux proteins are not homogenous among different tumor cell types which can explain the differential responses to the P-gp inhibitory effect of quercetin in T47D and MDA-MB-231 cells compared to MCF-7 [56–58].

## 5. Conclusions

In conclusion, despite the potent vascular protective effect of quercetin against doxorubicin-induced vascular toxicity, it might seriously attenuate its anticancer potencies. Quercetin and quercetin-rich dietary vegetables/fruits should be used with high care during the cycles of doxorubicin treatment. The strong antagonistic interaction between quercetin and doxorubicin in different breast cancer cell lines might be attributed to the strong antioxidant activity of quercetin, which abolishes the generation of doxorubicin-related reactive oxygen species with subsequent weaker tumor cell killing effect.

## Figures and Tables

**Figure 1:** Impaired vascular reactivity (contraction/relaxation) of aortic rings due to incubation with DOX. Freshly isolated aortae were incubated with serial dilutions of DOX and their responsiveness to PE (a, c) and Ach (b, d) were assessed in isolated organ bath. Data is presented as mean ± SD; *n* = 6-8. ^∗^Significantly different from the control group at *p* < 0.05.

**Figure 2:** Protective effects of quercetin against DOX-induced impaired vascular reactivity (contraction/relaxation) of aortic rings. Freshly isolated aortae were incubated with 10 *μ*M of DOX with serial concentrations of quercetin (a, c) and compared to its exposure to serial concentrations of quercetin alone (b, d). Aortic rings' responsiveness to PE (a, b) and Ach (c, d) were assessed in isolated organ bath. Data is presented as mean ± SD; *n* = 6-8. ^∗^Significantly different from the control group at *p* < 0.05. ^#^Significantly different from the DOX-treated group at *p* < 0.05.

**Figure 3:** Vascular ROS scavenging activity of quercetin against DOX-induced ROS in situ. Control (C), DOX (10 *μ*M)-treated (D), DOX (10 *μ*M)+quercetin ((10 *μ*M)-treated (DQ10), or DOX (10 *μ*M)+quercetin ((100 *μ*M)-treated aortic rings (DQ100) were incubated with DCF fluorescent dye and fluorescent units were compared. Data is presented as mean ± SD; *n* = 6. ^∗^Significantly different from control group at *p* <0.05; (#): significantly different from the DOX-treated group at *p* < 0.05.

**Figure 4:** The effect of quercetin on the cytotoxicity of DOX in MCF-7 (a), MDA-MB231 (b), and T47D (c) cell lines. Cells were exposed to serial dilution of DOX (●), quercetin (○), or DOX+Que combination (▼) for 72 h. Cell viability was determined using SRB assay. The intracellular/total concentrations of ROS were determined using CMFDA fluorescent dye after 1 h (d) and 24 h (e, f) of exposure to DOX, quercetin, their combination, and TBHP as a positive control. Data is presented as mean ± SD; *n* = 6. ^∗^Significantly different from the control group at *p* < 0.05.

**Figure 5:** Effect of DOX, quercetin, and their combination on the cell cycle distribution of MCF-7 (a), MDA-MBA231 (b), and T47D (c). Cell cycle distribution was measured by using DNA content flow cytometry analysis after PI staining and different cell phases were plotted as percentage of total events. Data is presented as mean ± SD; *n* = 3. ^∗^Significantly different from the control group at *p* < 0.05.

**Figure 6:** Apoptosis/necrosis assessment in T47D breast cancer cells after exposure to quercetin (b), DOX (c), and their combination (d) for 24 h in comparison to control cells (a). Cells were stained with annexin V-FITC/PI and different cell populations were plotted as percentage of total events (e). Data is presented as mean ± SD; *n* = 3. ^∗^Significantly different from the control group at *p* < 0.05.

**Figure 7:** Assessing the interaction properties of quercetin with the two subunits of P-gp efflux pump (P-gp ATPase and substrate binding site) using sodium vanadate (Sod. vanadate) and verapamil (VRP) as positive controls, respectively (a), and compared to the nontreated control (NTC). The intracellular concentrations of the fluorescent P-gp substrate (rhodamine) was measured after treating MCF-7 cells (b), MDA-MB-231 cells (c), and T47D cells (d) for 24 h with serial concentrations of quercetin or verapamil and compared to rhodamine alone. Data is presented as mean ± SD; *n* = 6. ^∗^Significantly different from NTC at *p* < 0.05. ^#^Significantly different from the Rho group at *p* < 0.05.

**Table 1:** Effect of quercetin on the cytotoxicity parameters of DOX in breast cancer cell lines. IC_50_s and resistance fraction (*R* values) were calculated using *E*_max_ mathematical model as shown in Materials and Methods. IC_50_ is the concentration of a drug or drug combination killing 50% of the cells, and *R* value is the percentage of cell resistance to drug/drug combination at the highest possible concentration of exposure.

	MCF-7		MDA-MB231		T47D	
	IC_50_ (*μ*M)	*R* value (%)	IC_50_ (*μ*M)	*R* value (%)	IC_50_ (*μ*M)	*R* value (%)
DOX	0.35 ± 0.1	4.3 ± 0.8	0.8 ± 0.02	2.7 ± 0.3	0.7 ± 0.09	5.8 ± 0.9
Quercetin	97.7 ± 7.2	6.2 ± 0.3	38.4 ± 4.8	4.2 ± 0.7	78.4 ± 11.9	6.1 ± 1.1
DOX+Que	0.8 ± 0.1	3.1 ± 0.2	0.8 ± 0.01	1.9 ± 0.9	0.36 ± 0.05	0.4 ± 0.1
CI value	Antagonistic/3.16		Antagonistic/2.04		Additive/0.96	

## Data Availability

Raw data and detailed data analysis files are available upon request from the corresponding author (ahmedmalabd@pharma.asu.edu.eg).
